# Augmented Reality-Centered Position Navigation for Wearable Devices with Machine Learning Techniques

**DOI:** 10.1155/2022/1083978

**Published:** 2022-04-07

**Authors:** G. K. Kamalam, Shubham Joshi, Manish Maheshwari, K. Senthamil Selvan, Sajjad Shaukat Jamal, S. Vairaprakash, Musah Alhassan

**Affiliations:** ^1^Department of Information Technology, Kongu Engineering College, Perundurai, Erode, Tamil Nadu, India; ^2^Computer Engineering, SVKM'S NMIMS MPSTME, Shirpur Campus, Shirpur, India; ^3^Department of Computer Science and Applications, Makhanlal Chaturvedi National University of Journalism and Communication, Bhopal, Madhya Pradesh, India; ^4^Prince Shri Venkateshwara Padmavathy Engineering College, Chennai, Tamil Nadu, India; ^5^Department of Mathematics, College of Science, King Khalid University, Abha, Saudi Arabia; ^6^Department of ECE, Ramco Institute of Technology, Rajapalayam, Tamil Nadu, India; ^7^University of Development Studies, Electrical Engineering Department, School of Engineering, Nyankpala Campus, Nyankpala, Ghana

## Abstract

People have always relied on some form of instrument to assist them to get to their destination, from hand-drawn maps and compasses to technology-based navigation systems. Many individuals these days have a smartphone with them at all times, making it a common part of their routine. Using GPS technology, these cellphones offer applications such as Google Maps that let people find their way around the outside world. Indoor navigation, on the other hand, does not offer the same level of precision. The development of indoor navigation systems is continuously ongoing. Bluetooth, Wi-Fi, RFID, and computer vision are some of the existing technologies used for interior navigation in current systems. In this article, we discuss the shortcomings of current indoor navigation solutions and offer an alternative approach based on augmented reality and ARCore. Navigating an indoor environment is made easier with ARCore, which brings augmented reality to your smartphone or tablet.

## 1. Introduction

Tools such as maps and compasses have helped travellers since ancient times. They had an important role in the daily lives of the people of the past. Without the help of these tools, the time to reach their destination would have been extended by a large amount. In modern times, people rely on the power of technology for navigational purposes. With the growing popularity of smartphone technology, smartphones have become one of the prominent devices of the modern era. Almost all people are equipped with a smartphone these days. They have inbuilt applications such as Google Maps, which uses the GPS technology for facilitating outdoor navigation. The accuracy of the outdoor navigation provided by this kind of application is fairly high, but when the same applications are used in the indoor environment, the accuracy is extremely low. Buildings with complex internal environments such as universities, malls, and industries are hard to navigate for the people who are visiting for the first time. Therefore, reaching their destination becomes a time-consuming process. The greatest challenge for navigating such environments is to guide the people to their destination in the most optimal manner and with the highest possible accuracy.

Walking instructions are superimposed over real-world streets using the augmented reality navigation tool. The map would be shown using a smartphone camera and would indicate us where we were and when we needed to turn left or right, or just keep going straight.

Because GPS signal is readily attenuated in a complex inside environment, it is recommended that alternate indoor location technologies be used instead of GPS. It might be divided into five main categories based on the baseband and theory of positioning technology.

1. Positioning Technology Based on Ultrasonic: the ultrasonic positioning system is constituted of a large rangefinder and various electronic labels [1]. In order for the system to function properly, the rangefinder must deliver a signal. Electronic labels, after receiving the signal from the rangefinder, send the same signal back to the rangefinder to confirm receipt of the label. This procedure may be used to compute the distance between two points. Ultrasonics, on the other hand, can only be employed in a particular limited region due to the attenuation that occurs throughout the propagation process.
2. Second, infrared light is used for positioning purposes because its wavelength is halfway between radio and visible light [2], which allows it to be used in both indoor and outdoor applications. For example, active badges use an infrared light localization system to locate the wearer. In this method, an electronic label will be automatically placed on a target, and the label will emit infrared light at regular intervals. The signal will be received by the receiver, which will be positioned inside, and the signal will be sent to a database over the Internet. [3] After then, it is possible to compute and acquire the location. Infrared light, on the other hand, may be obstructed by objects such as glass, a wall, or a chair. Furthermore, the valid transmission distance would be restricted, and the system itself would be complicated.
3. Ultra-Wideband Positioning Technology: ultra-wideband (UWB) positioning technology offers various benefits, including fast transmission speed (up to 1000 Mbps), low-power consumption, wide penetration, and the absence of a carrier [4], so it is more precise than the other technologies listed before.

Various techniques such as Bluetooth, Wi-Fi, RFID, and computer vision were implemented to tackle the issue of low accuracy [3, 5]. These techniques were able to increase the accuracy of indoor navigation, but they had their drawbacks [4, 6–11]. Augmented reality (AR) is a reality-altering technology that is under rapid development [1, 2, 12–24]. AR enables virtual objects to be perceived along with real-world objects. There are several software development kits (SDKs) that make the development of the application easier. Some of the specific SDKs for the development of AR applications include ARCore, ARKit, and Vuforia. ARCore enables AR development for android devices, and ARKit enables AR development for Apple's iOS.

## 2. Background

### 2.1. Previous Technologies

Bluetooth technology focuses on using beacons for improving the accuracy of indoor navigation [4, 6–11]. Bluetooth low energy (BLE) technology provides the necessary setup by mounting several beacons that send signals, which is used to determine the location in an indoor environment [3, 5]. These beacons are radio transmitters that can emit signals in the range of 10 to 30 meters. They provide an accuracy of up to one meter. Based on the detected beacon, it is also possible to determine the current floor where the user is at.

Wi-Fi technology is similar to Bluetooth technology, but instead of using beacons, it uses Wi-Fi hotspot points to calculate the position of the device [23]. The received signal strength indication (RSSI) helps in determining the position of the user. The accuracy of this method is 5 to 15 meters, which is far lesser compared with the beacon method [24]. The distance is calculated using the latitude, longitude, and relative position of the device with each Wi-Fi access point.

The radiofrequency identification (RFID) method uses the information saved into a tag that can track in an indoor environment. It is most commonly employed in the logistics sector where they have to keep in track of their materials [25]. This simulation is carried out in five critical performance metrics to categorize and classify the damaged rice plant and decide the classification of the plant. The passive tags are not provided with any energy, and they obtain power from the readers. However, the other tags are provided with an energy storage component [26].

### 2.2. Technology Limitations

The abovementioned technologies have greatly helped in increasing the accuracy of indoor navigation, but they have their limitations too. Bluetooth beacons have greater accuracy compared with Wi-Fi access points, but the downside to this accuracy is that it is directly proportional to the number of beacons used. Mounting beacons over a small area such as an office is easy and cost-effective, but when it comes to a larger structure such as universities, it becomes impractical [26]. The problem with the Wi-Fi access points is not only its accuracy but also the fact where failing to establish a connection to the device or a delay in the connection may result in errors and false mapping of the user's position. The RFID technology may be suitable for implementing in buildings such as a warehouse, but it is not suitable for implementing in universities or malls. For higher performance and accuracy, we can use the active tags, but they are very costly. Moreover, a large number of tags are required to cover such a huge area. Passive tags can be used instead of active tags, but the range and efficiency of these tags pale in comparison with that of the active tags [27].

### 2.3. Augmented Reality and ARCore

In 1968, a system known as the “*Sword of Damocles*” was introduced, which would later become the predecessor for the reality technologies. Augmented reality (AR) specializes in overlaying the real-world environment with virtually generated objects. The goal of AR is to provide the most clear and accurate representations where the user finds it hard to differentiate the virtual augmentations that are being applied [26]. AR is employed in various applications, including game development, military training, simulations, design, and entertainment [28]. The increasing popularity of the AR technology has led to the rise of several SDKs, which support the development of the AR applications. Vuforia, ARCore, and ARKit are some of the SDKs for developing AR applications. Vuforia has a recognition feature for identifying various visual objects and environments [29]. Local storage or cloud storage can be used to enable the recognition feature. ARKit was developed by Apple, which can be enabled from iOS 11 and later versions. It supports the creation of AR applications for iPad and iPhone.

ARCore was developed by Google for building AR applications. It works only for a specific set of devices, but the number of supported devices is increasing steadily. There are three key technologies in ARCore that allow the integration of the virtual and physical world using the device's camera.

1. Six degrees of freedom are provided, which enables the device to realize the current position and track accordingly with respect to the world coordinates.
2. The understanding of the environment enables a device to track the position of the planes such as the floor plane and the top flat surface of pieces of furniture. It can also detect the size of such surfaces.
3. The light estimation feature enables the device to detect and analyze environmental lighting and provides various methods to act upon it.

## 3. Literature Survey

Austin Corotan et al. [12] implemented an augmented reality system for the purpose of indoor navigation. They created an app that acted as a controller and could also perform sensing operation. Arduino Uno had powered their robot. The robot had a smartphone mounted on it to navigate automatically and carry out localization operations. The autonomous navigation had three major aspects, which include object detection, localization, and routing. Q-learning algorithm was used for optimally planning the route and the blueprint, of the navigation path. They used a parser that could split a floor map into smaller states. They solved the localization issue using the motion tracking system of ARCore along with a scaled blueprint.

Anthony Francis et al. [13] implemented a long-range indoor navigation using PRM-RL. They implemented the system by training a planner, which is independent of the environment, creating a small road map for the planner followed by data query, generating trajectories, and data execution. They have evaluated the performance with the basic blueprints of the floor layers and using the SLAM maps. They have analyzed the various threshold values that were obtained from the robot and set variable velocities to test the performance. The numerical data of the physical experiments have been tabulated. The simulation environment was created from the real-world environment perspectives, and the metric maps were derived from them.

Michel et al. [14] implemented a system for precise identification of attitude for indoor navigation using AR and smartphones. The device's accelerometer, magnetometer, and gyroscope were all used in conjunction to assess the variation in attitude. It is possible to achieve a defined quaternion and a compensated drift. They verified the accuracy of the recorded measures using iPhones and Android devices to take the measurements. They varied the sampling rate of the sensors and tested out the associated algorithms for precision according to sampling rates. Their tool and experimental protocol allowed them to confirm the parameter values that yield the best results.

Al Rabbaa et al. [15] implemented a multisensory application with a simplified cognitive effort requirement. The cyclical process involved three stages: ideation, user interface, and user experience. Using place note SDK, the world was scanned using the camera of an iPhone. The varying depths of the surrounding space were calculated, and 3D point clouds of the horizontal and vertical planes were represented. The multisensory experiences were tested with a few human participants, and their feedback was used for further improvement of the system.

## 4. Proposed System

The goal of the system is to overcome the limitations of the previous technologies (Section 2) using AR technology for indoor navigation. AR technology development has been made simpler because of the latest SDKs. It provides a simple and inexpensive solution for navigational purposes.

Because they have long-term consistent precision, using accelerometers and magnetometers to get orientation is a smart long-term strategy. However, the difficulty is that they are subject to unanticipated external disturbances, which implies that they are unstable in the short run. Given that we cannot get an ideal orientation result just from a gyroscope, we use an accelerometer and a magnetometer to provide extra orientation information that may be used as a reference to correct the gyroscope mistake.

The getOrientation method on Android is used to determine one's location. There are two arguments to this function. The first value, *R*, is a rotation matrix, and the second value is an array of three floats to retain the output of the rotation matrix. We must first use the get rotation matrix function to get the rotation matrix before we can apply this method.

The following are examples of values [0]: when the smartphone is positioned horizontally, the azimuth is the angle of rotation around the z-axis, which represents the heading.

### 4.1. System Requirements

The application is focused on android mobile devices that can support ARCore. The list of supported devices has been provided by Google in their developer site under the supported device section. Software packages such as Android Studio and Unity are required for building the application along with the Android Gradle build support [29]. The level of the android package used should be at least 24 to support the application development. Android Studio 3.1 or later and Unity 2017.4.34f1 or later versions are necessary for importing and integrating ARCore into the project.

  The Linux Kernel: the Linux kernel is responsible for the majority of Android's system services. It also serves as a layer of abstraction between the hardware and the software stacks [1–3, 5, 17].
  Hardware Abstraction Layer (HAL): in layman's words, the Android hardware abstraction layer is the Linux kernel driver package that serves as an interface between the top layer and the lower layer, while hiding the implementation of low-level features. In other words, the hardware support is separated into two layers, one in the user space and another in the kernel area, each with its own set of capabilities. The rationale for this is because it is in accordance with the GNU License. Android Runtime: Android Runtime (ART) is an operating system environment that runs on Android devices. It was created by Google in 2013 as a test feature for the Android 4.4 operating system and released in 2015. Android 5.0 and following Android versions were the first to include the ART feature. As a formal runtime library, it took the place of the preceding Dalvik virtual machine in the Java virtual machine. ART can translate the bytecode of an application into machine code, which is a new virtual machine that is used by the Android operating system. When comparing Dalvik with ART, the most significant distinction is that Dalvik employs just-in-time (JIT) technology, whereas ART employs ahead-of-time (AOT) technology. The performance of the system, trash collection, application debugging, and performance analysis are all improved by ART.
  Native C/C++ Libraries: Android offers a number of C/C++ libraries that are native to the platform. The Android application framework allows developers to use the services provided by these companies. In addition to the fundamental C library, multimedia libraries that support a wide range of multimedia types, bitmaps and vector fonts, a 2D and 3-dimensional graphics engine, a browser, and database support are all included in the core libraries [5].

## 5. System Overview

The system comprises two modes of operation: user mode and admin mode. The admin mode allows access to the cloud storage for storing the navigational markers that are set to real-world environments. In this mode, the device scans its environment and acquires a basic understanding based on the detected points of interest (PoI). Once the required PoI is detected, the ground plane detection algorithm starts estimating the size and distance of the floor. The detected floor surfaces can now be superimposed with the virtual objects (navigational markers). These markers are then hosted to the cloud storage for later retrieval using the cloud anchors. Latitude and longitude coordinates along with the detected features are captured when a marker is placed and these data are stored such that there is no deviation of the marker placed in the real-world environment when the application is used at a later time.

The user mode is provided to the people who seek navigation within the complex indoor environment. When the user opens the application, the recent places that have been visited pop up to make the search easier. If the required destination is not displayed in the recent bar, it is possible to search for the destination manually. Following the selection of a destination point, the user interface changes to the augmented reality navigation interface. The device scans the surrounding area and compares the detected feature points with those previously recorded in the cloud. As soon as a match is identified, the navigational markers are presented, guiding the user to their location in the most efficient manner possible. The state of optimality is reached by analyzing the shortest route using the shortest route detection algorithm, which maps the points that are stored in the cloud and finds the shortest route with the *A*∗ algorithm [25]. When the user reaches their destination, the navigation interface jumps back to the home interface and the user is able to search for a new destination.

ARCore provides the ground plane detection, light estimation, and environmental understanding features, which play an important role in the implementation of this project. The ground plane detection algorithms are able to clearly define any flat surfaces such as the floor or tabletops, which have well-defined feature points. The light estimation allows to react to the instances of light that are available in the surroundings. It also enables the brightening up of the scene when a specific flag is triggered. The environmental understanding enables the device to identify the POI and then analyze the data to determine the type of object that is detected. Making use of these features, an interactive indoor navigation system is provided to efficiently reach the destinations inside a complex indoor environment.

## 6. System Design

The home interface of the mobile application is shown in Figure 1. From the home interface, the user mode and the admin mode are accessible. Selecting any of the destinations that are displayed in the recent bar would immediately display the user mode navigation interface. To improve the user experience, the switching of the interfaces was implemented with a smooth transition and different backgrounds were applied to the home interface. The unique destinations were provided with their own icons to make the process of finding them easier. The plane detection algorithm works when the camera of the device is focused on the ground. Since the user is unaware of this information, the user navigation interface provides a small animation indicating that the user should focus their device camera on the floor. When the user successfully completes this task, the detected planes are represented by a dot mesh on the floor. Based on the orientation of the device, it is able to identify the walls and other obstacles too, but there are no visual representations for them similar to the dot mesh of the ground.

As previously indicated, each indoor positioning method has its own set of advantages.

However, there are flaws in the system. Because of GPS signal propagation attenuation [17], the precision of locating technology based on GPS is inadequate. Positioning technique based on short-distance wireless communication has a limited coverage area because of its short range. If we wish to improve the precision of the system, more hardware will be necessary. In comparison with short-distance wireless communication, the positioning system based on Wi-Fi has a greater range covered and a more acceptable level of accuracy [8]. Because there is no accumulated deviation, it is excellent for long-term use and servicing. However, the accuracy of the system is dependent on the distribution of existing wireless network access points, unrelated external noise, and the RSSI database, all of which significantly raise the cost and restrict the range of applications. The inertial sensor-based positioning technology is extensively used since it is inexpensive in cost, compact in size, and capable of autonomous placement. However, because of the accumulating deviation, it cannot be used for an extended period of time.

It is the primary objective of this thesis to develop indoor positioning technologies that are wide, continuous, autonomous, and highly effective in order to implement a positioning system with an inertial sensor and a wireless signal transmission.

As the Internet and the Internet of things (IoT) have grown in popularity, they have brought about several changes in our lives. According to a forecast issued by IHS iSuppli [20], the total number of smartphone and tablet users in the world will reach 1.03 billion by the end of the year 2015. Worldwide, there will be more than 4 billion smartphone users by the end of this year, and everyone will be able to use this “Palm-Sized PC” to connect to the Internet.

It is the autonomy and continuity of the inertial sensor that distinguish positioning technology based on this sensor. An accurate result may be obtained in a short period of time because of the tiny size of the hardware, its cheap cost, its endless uses, and the fact that it is not affected by external signals. However, the problem of deviation buildup has not yet been resolved. Wi-Fi-based positioning technology has the potential to be broadly diffused inside and is well suited for large-scale positioning applications.

There are few instances where the system is not able to correlate the data stored in the cloud and the data that are currently being detected by the device camera. This may happen when there are insufficient feature points or when there is a problem of establishing a connection to the cloud storage. The problem of insufficient feature points can be easily solved when the device is moved around a little and camera is focused on adjacent areas as well. The problem of establishing a connection depends on the available network speed and coverage. This device and the location-specific issue can be resolved if the user has appropriately secured and maintained a stable connection.

The dataflow model of a sophisticated indoor navigation system is shown in Figure 2, which represents the sequence of execution and the various components that are involved. The project involves a simplified system where ARCore is the heart of the system and the cloud storage is the database used. The detection and analysis algorithms are integrated into the ARCore such that there are no separate calls to the function. The data stored in the cloud are not related to the destinations rather it is the position data of the markers placed in the real-world environment.

## 7. Experimental Setup

To monitor a person's whereabouts, location-based services make use of the GPS technology included in a smartphone, provided that the individual has given their consent. The programme can detect a smartphone user's position down to the street address once they have opted in, eliminating the need for human data input. We conducted an experiment to test the accuracy of the system. The markers were limited to a single floor, and they were set to point to the various laboratories available in that floor. A white-tiled surface covered the entire region of the floor along with glass walls and doors that bounded the laboratories. Every laboratory was registered as a destination in the mobile application. The two participants were asked to choose different destinations, and they started navigating simultaneously. Even though every location of the floor was almost identical, the system was able to detect the markers that were placed in the admin mode and were properly rendered in the user mode. They were successfully able to reach their destinations without any problems. The results have confirmed the localization, positioning, and rendering capabilities of the system in a small-scale environment.

## 8. Discussion and Results

In comparison with the previous technologies mentioned in Section 2, augmented reality provides a simpler method for indoor navigation. ARCore has greatly simplified the process of developing the AR application and has provided various methods that are well suited for acquiring data from the environment. In addition to being simple to develop and implement, it is also an inexpensive solution where there is no requirement of hardware to produce signals for positioning and tracking within the indoor environment. The interface provided by AR is very interactive, and the user experience is greatly improved compared with the earlier technologies. The accuracy that we obtained by carrying out the above experiment was also found to be higher compared with the previous technologies.

The accuracy comparison of the various technologies used for indoor navigation is shown in Figure 3. From the above representation, it is clearly evident that the accuracy of GPS is the lowest for indoor navigation. This is due to the fact that the reception of the satellite signal is very low in the indoor environment. Wi-Fi has a higher accuracy compared with GPS as there are hotspot setups in various locations within the indoor environment. The received strength of the signal helps in the location estimation of the navigating device.

The localization method of Bluetooth beacons is the same as Wi-Fi, but it offers a higher level of accuracy. The highest accuracy is offered by the AR technology in combination with ARCore. The AR technology is not based on signals rather it focuses on observing the indoor environment and uses the data that are stored in the cloud for positioning and localization.

Because they have long-term consistent precision, using accelerometers and magnetometers to get orientation is a smart long-term strategy. However, the difficulty is that they are subject to unanticipated external disturbances, which implies that they are unstable in the short run. Given that we cannot get an ideal orientation result just from a gyroscope, we use an accelerometer and a magnetometer to provide extra orientation information that may be used as a reference to correct the gyroscope mistake.

The getOrientation method on Android is used to determine one's location. There are two arguments to this function. The first value, *R*, is a rotation matrix, and the second value is an array of three floats to retain the output of the rotation matrix. We must first use the getRotationMatrix function to get the rotation matrix before we can apply this method.

There are four arguments to this function: *R* denotes the rotation matrix, and *I* denotes the same as *R*. Gravity and geomagnetic fields may be measured with relative ease using accelerometers and magnetometers. The following are examples of values [0]: when the smartphone is positioned horizontally, the azimuth is the angle of rotation around the z-axis, which represents the heading.

Earlier, navigation technologies were used to work on a two-dimensional frame. The navigation was only based on the *X* and *Y* dimensions. The maps were represented as a planar surface, and the position of the device was represented by a dot on that map. The third dimension for navigation was introduced by technologies such as AR and computer vision.  Table 1 shows the various navigation technologies along with their dimensional characteristics, accuracy, and usability. AR provides the highest level of usability due to its super-friendly user interface and easy-to-understand navigation. The difficulty associated with visual recognition and SLAM technology is because of the complexities in mapping the device location and positioning it accordingly.

After that, we posed questions on the significance of battery usage as a feature of an app. The following questions were asked: how often do you charge your phone? Do you believe that the power consumption of a software programme is significant? If there is an app with the same purpose and has slower power usage, would you replace the existing one with it? Which of the following, in terms of accuracy and power usage, do you believe is most important? The result is that 41.7 percent of participants charge their phone more than twice per day and 54.1 percent of participants charge their phone once or twice per day. Only one person charged their phone more than once every day and that individual was the only one. More than 90 percent of those who took part in the survey believed that power consumption was important, but that increased consumption was acceptable if the application was extremely useful. Participants agreed that accuracy was more essential than power consumption in a navigation app, but they said they would replace the existing app with a lower power consumption application that performs the same purpose as the current app.

The question set included questions such as “What do you think about an indoor navigation application?” and “What do you think about an indoor navigation application?” to gauge people's expectations for an indoor navigation application. Were you ever in the position where you needed to use an indoor navigation application? When making a decision to use an indoor navigation application, what factors would you consider? What do you think is a reasonable pricing for the app? The findings revealed that none of the participants had ever used an indoor navigation app previously, but that they were all enthusiastic about the prospect of doing so. When it comes to using such an application, the majority of individuals believe that accuracy and convenience of use are both significant considerations. The price that was acceptable was less than $5.

Finally, according to the survey results, the majority of respondents have not used an interior navigation application, but all of them are interested in doing so, indicating that the future of this app is bright. The accuracy of a navigation application is also very significant to users, as we discovered throughout our research! The usage of electricity was also considered 40 to be significant. Users favoured a low-power consumption application over an application that performed the same job but used a large amount of battery power.

The AR technology is under rapid development, and updates are being constantly released to improve the efficiency. The reality-based technologies have become very popular in recent years due to their rich user experience. These technologies are able to produce an environment where the border between virtuality and reality is broken down and it became harder to differentiate from one another. It enables a scenario where the virtual objects can be brought into the real world or the real-world objects can be brought into the virtual world. It makes the user to experience a world that is fundamentally different from what they are normally used to. These technologies have the potential to unlock unlimited possibilities, which could be incorporated into every existing field of work.

They are currently being used in a wide range of fields such as video game development, military training, vehicle simulations, and component design and are considered to be some of the top technologies of the future. The complexity and efficiency comparison of the various technologies used for indoor navigation is shown in Figures 4 and 5.

## 9. Conclusion and Future Evolution

The solution that has been provided here is an inexpensive and convenient indoor navigation system that does not require any additional hardware. This system was particularly checked for effectiveness within a university campus, and the results proved to be satisfactory. The AR-based navigation system provided an immersive experience to the users from the start of their route till they reached their destination. This immersive experience can be further improved by integrating a voice support, enhancing the details provided during the navigation, and adding fun features such as character guides to the navigation system. This indoor navigation system uses common cloud storage for holding all the markers that are placed in the real-world environment. However, it is inefficient while implementing this project in a large scale across various malls and universities.

Fortunately, creating distinct storage locations for each different internal environment helps alleviate this issue, which prevents a memory overflow from occurring when the device attempts to retrieve the marker information. Further improving the system by allowing for faster recovery from storage and smoother rendering on the device's screen would be a significant improvement. It would be possible for the user to traverse the interior environment by integrating the abovementioned voice assistance system, character guiding system, and natural language processing (NLP) system into one system. The usage of natural language processing (NLP) would be a fantastic addition to the system since it would enable users to simply get their destination using voice input. English is one of the world's most widely spoken languages, with over a billion speakers. As a result, the majority of NLP systems are designed to work with the English language. This kind of technology, however, would be useless to the general public since they are not familiar with languages other than their own tongue. A significant improvement in user experience and enhanced utility for a variety of communities might be achieved by expanding the NLP system to accommodate numerous local languages as it develops.

The major focus of future development of indoor navigation system would be to increase the efficiency of the system's marker tracking and positioning along with efficient storage and retrieval. The system should not only cover the premises of a single university, but it should be able to detect the location of any indoor environment that is integrated into the system. The position of the building is determined from the latitude and longitude coordinates obtained using the GPS technology. This information is relayed to the server, which calls the appropriate marker information from the cloud storage corresponding to the detected indoor environment. Thus, the system would be able to guide the users to their destination in various indoor environments simultaneously and efficiently.

Another issue with our system is that the position of the initial point is chosen by the user, which means that if the point is picked incorrectly, all subsequent location information, with the exception of the path's shape, would be incorrect. This is one of the faults with our system. Finding a solution to that challenge is one of the potential future expansions of this study.

We developed an interior navigation system on the Android platform to make people's lives more convenient and to assist them in the event of an emergency. Our objective was to make the system as accurate as possible while still using as little electricity as possible. To achieve our aim, we developed a sensor fusion technique that used the accelerometer, magnetometer, and gyroscope that are all located inside the smartphone, and we integrated the data from these sensors to get the high-accuracy heading. Afterwards, we used a step sensor, which was low in power consumption, and Kim's method [23] to determine the distance travelled over a period of time. To keep track of the user's location, a dead reckoning method is used. The following are the characteristics that our system has accomplished in its present condition.

1. An Application for the Android Smartphone Platform. Due to the fact that we developed our system only on the sensors that are already present in the Android smartphone, we did not need to include any additional sensors or technologies, such as Wi-Fi. A smartphone does not have to be costly, and they are frequently used, which makes the application feasible and accessible to the general people, as well as to researchers.
2. Make Use of the Sensors. Our system does not rely on a single sensor to function properly. We developed a sensor fusion system that used a variety of sensors and applied a filter to provide a very accurate outcome.

Furthermore, we need further tests to demonstrate the effectiveness of our method. Using our multi-sensor navigation system, we were able to compare the performance of a single sensor with our multi-sensor system.

Ongoing research will compare the performance of our system with the performance of other technologies or applications in the same field.

In addition, we need extra features to make the programme more user-friendly. We wish to include a variety of relevant technologies into our application and provide consumers with more possibilities. We also need to make improvements to the map functionality. Currently, users may only use maps from their local sources, which imply that they must also be aware of the size of the map in question. We may be able to construct a map warehouse in the future to store indoor maps and their scales. All that would be required of users would be to download the map from the warehouse. A user-generated indoor map of the warehouse might also be uploaded to the warehouse.

Finally, we need more test data to correct the algorithm in our system. We conducted all of our trials inside the confines of the institution, which seems to be inadequate. As part of our future effort, we will submit our application to the app store and invite additional users to assist us in testing the overall functioning of our platform.

## Figures and Tables

**Figure 1:** Mobile application interface.

**Figure 2:** Dataflow representation.

**Figure 3:** Accuracy of navigation technologies.

**Figure 4:** Complexity of navigation technologies.

**Figure 5:** Flexibility of navigation technologies.

**Table 1:** Comparison of navigation technologies.

Name	Type	Accuracy	Setup (1 = easy, 5 = hard)	Usability
Bluetooth beacons	2D	3–8 m	3	3
Compass-based	2D	5–10 m	4	1
Apple indoor maps	2D	4–8 m	3	1
Ceiling antennas	2D	10–50 cm	5	2
GPS	2D	5–15 m	1	3
Visual recognition/SLAM	3D/6DoF	10–30 cm	4	1
Markers/QR codes (AR)	3D/6DoF	5–15 cm	1	4

## Data Availability

The data that support the findings of this study are available on request from the corresponding author.
